# Differential expression of circulating miRNAs as a novel tool to assess BAG3-associated familial dilated cardiomyopathy

**DOI:** 10.1042/BSR20180934

**Published:** 2019-03-15

**Authors:** Carlos Zaragoza, Marta Saura, Ignacio Hernández, Rafael Ramirez-Carracedo, Francisco García-García, Jose L. Zamorano, Alipio Mangas, Rocio Toro

**Affiliations:** 1 Cardiology Dept, Univ Francisco de Vitoria, School of Medicine/Hosp Ramón y Cajal Res Unit (IRYCIS), Madrid, Spain; 2 Dept of Systems Biology (Physiology), Univ de Alcalá, School of Med (IRYCIS), Alcala de Henares, Madrid, Spain; 3 Bioinfomatics and Biostatistics Unit, Principe Felipe Research Center, Valencia, Spain; 4 Cardiology Dept, Univ Hosp Ramón y Cajal (IRYCIS), Madrid, Spain; 5 Univ Puerta del Mar, School of Medicine, Cadiz, Spain

**Keywords:** BAG3, familial dilated cardiomyopathy, microRNA

## Abstract

A new familial dilated cardiomyopathy (FDCM) was found related to mutations in *BAG3* gene. MicroRNAs (miRNAs) represent new targets of FDCM, although no studies have assessed clinical association between Bcl2-associated athanogene 3 (BAG3)-related DCM and miRNAs. Here, we studied whether a clinical association between BAG3-related FDCM and circulating miRNAs may have diagnostic and prognostic value in a small cohort of familial related individuals carrying a BAG3 mutation (BAG3+) and/or diagnosed of dilated cardiomyopathy (DCM) (DCM+). The analysis of 1759 circulating miRNAs showed significant differences between BAG3+ and BAG3- individuals for miRNAs mir-3191-3p, 6769b-3p, 1249-ep, 154-5p, 6855-5p, and 182-5p, while comparisons between BAG3+/DCM+ versus BAG3+/DCM- were restricted to miRNAs mir-154-5p, 6885-5p, and 182-5p, showing significant correlation with systolic and diastolic blood pressure, A wave, left atrium length, and left atrium area. Additionally, when stratified by gender and age, miRNAs were statistically correlated with critical parameters, including left ventricle ejection fraction (LVEF) and ventricular diameter, in women and young men. Likewise, 56% of BAG3+/DCM+, significantly co-expressed mir-154-5p and mir-182-5p, and a slight 4% did not express such combination, suggesting that co-expression of mir-154-5p and mir-182-5p may potentially show diagnostic value. Further studies will require long-term follow-up, and validation in larger populations.

## Introduction

Bcl2-associated athanogene 3 (BAG3) is a 575 amino acid anti-apoptotic protein that is constitutively expressed in the heart, skeletal muscle, and some types of cancers. BAG3 works as a co-chaperone wit Hsc-70 facilitating the removal of misfolded and degraded proteins, and inhibits apoptosis by interacting with Bcl2 and maintaining the structural integrity of the Z-disk in the muscle [1,2]. Functional studies revealed that some forms of familial dilated cardiomyopathies (FDCMs) are related to BAG3 mutations with impaired Z-disc assembly and sensitivity to stress-induced apoptosis [3] proposing that myofibrillar integrity under mechanical stress is maintained by the complex BAG3–Hsc70, since Hsc70 regulates the chaperone-dependent E3 ligase CHIP [4,5].

BAG3 mutations related to FDCM were first described in individuals from the same familial group with diffuse fibrosis and sudden death [6]. The relevance of BAG3 in the etiology of dilated cardiomyopathy (DCM) arise from studies in which the levels of BAG3 in the heart of patients with advance heart failure were significantly reduced, suggesting that BAG3 may represent a critical component to prevent heart failure [7]. We have recently identified a rare variant causative of FDCM, detecting a novel frameshift (p.H243Tfr*64) genetic variation in BAG3 that is segregating in all affected family members, and it correlates with a severe phenotype of DCM [8].

MicroRNAs (miRNAs) are small non-coding RNA (20–25 nucleotides) that play a key role in gene regulation. In recent years, miRNAs have emerged as epigenetic regulators in the development and physiology of the cardiovascular system [9], and deregulation of miRNA expression has been directly associated with the pathophysiology of a large number of cardiovascular diseases [10,11]. Circulating miRNAs have been studied as mediators in intercellular communication and as potential biomarkers of disease [12,13] including myocardial infarction, coronary artery disease or heart failure [14,15]. Nevertheless, the role of circulating miRNAs as biomarkers of familial DCM are scarce [16]. We aim to analyze the association between circulating miRNAs and familial DCM caused by the mutation on BAG3 gene.

## Methods

### Population selection

The study has been performed in accordance with the ethical standards laid down in the 1964 Declaration of Helsinki and its later amendments such as the specific national laws. The study was approved by the ethics committee from the University Hospital Puerta del Mar, Cádiz, Spain. Written informed consent was obtained from all individuals included in the study. The study population included 44 BAG3 wild-type patients (20 DCM- and 21 DCM+), and 21 BAG3 mutation carriers (14 DCM+ and 7 DCM-), all of which belonged to the same family to avoid selection bias, except two independent healthy controls.

### Clinical presentation

Detailed clinical data was obtained from each subject, including family history, age of presentation, initial symptoms of HF, and physical examination, as we described [8]. Diagnostic criteria were evaluated by using 12-lead electrocardiogram (ECG), transthoracic echocardiography, tissue Doppler imaging, and ECG-Holter monitoring, when appropriate, as previously shown [8]. We have defined phenotypically positive those patients who exhibited left ventricle ejection fraction (LVEF) levels less than 50% and/or telediastolic left ventricle diameter larger than 55 mm.

### Sequencing

About 5 ml of peripheral blood samples were collected in PAXgene RNA tubes and stored at −80 °C before use. Total RNA was isolated using the PZXgene Blood miRNA kit according to manufacturer’s instructions (Quiagen), and quantified by spectrophotometry (Nanodrop). Quality control and integrity of samples were tested using the Agilent 2200 tapstation system (Agilent technologies). After that, we generated ultra-sequencing library preparation solutions with the NEXTflex Small RNA sequencing kit V2 (Bioo Scientific Corp) compatible with Illumina Platforms, by using 15 cycles of amplification. miRNAs were selected by size (152–154 bp), and sequenced (75 cycles) (Illumina NextSeq500) with the NextSeq 500/550 High Output Kit v2 (Illumina). Samples were read 50 times/run.

### Validation by quantitative real-time PCR (qRT-PCR)

Specific miRNAs were validated by quantitative real-time PCR. First, RNA was reverse transcribed, and the corresponding cDNAs were used as templates in Real Time PCR assays with specific PCR primers for each miRNA by using the SYBR PCR Master Mix (Thermo Fisher) on a 7900HT Fast Real-Time PCR System (Thermo Fischer). Relative expression levels were calculated with the 2-ΔΔct relative quantification method as previously described [17].

### Data analysis

We explored gene expression data by Principal Component Analysis and Clustering methods [18]. We filtered miRNAs without counts for all samples. miRNA-Seq data were normalized using Trimmed Mean of M values [19] and analyzed from the Bioconductor package *edgeR* [20], fitting a Negative Binomial Generalized Linear Model where design matrix included one factor for all experimental groups: BAG3-/DCM-, BAG3+/DCM+, BAG3-/DCM+, BAG3+DCM-. Conventional multiple testing *P*-value correction procedure proposed by Benjamini–Hochberg was used to derive adjusted *P*-values. Clustered heat map was performed as described [21].

The Pearson coefficient of correlation (*r*) was used to measure the linear correlation between selected miRNAs and clinical parameters. Only correlations with *r* > 0.4 with *P* values < 0.05 were considered.

Receiver Operating Characteristic (ROC) and the area under the ROC curves (AUC) were used to measure the performance of using combination of selected miRNAs to forecast disease [22].

## Results

### Clinical features of the members included in the study

Our study included a seven-generation Spanish family suffering from familial DCM, as previously reported [8]. A schematic representation of the study is shown (Figure 1A). Twenty-one members positive for a mutation in BAG3, were broken down into DCM+ (*n*=14), or DCM- (*n*=7) patients, and 44 BAG3 negative mutation carriers (DCM+ (*n*=21), and DCM-(*n*=20) (Table 1).

**Figure 1:** Schematic representation of the population study and miRNA distribution (**A** and **B**) Schematic representation of the study design, showing the strategy used to find the corresponding miRNAs of the study. (**C**) Clustered heat map of the differentially expressed miRNAs in the population study.

**Table 1:** Clinical and echocardiography features from population of the study

	BAG3-/DCM-N:20	BAG3-/DCM+N: 21	BAG 3+/DCM+N:14	BAG3+/DCM-N:7
**AGE**	40.92 ± 15.47	38.86 ± 14.68	45.21 ± 10.00	26.29 ± 17.43
**SEX (male%)**	10	11	10	3
**WEIGHT (kg)**	71.29 ± 14.66	74.88 ± 19.13	86.29 ± 15.22	58.00 ± 14.97
**HEIGHT (cm)**	168.92 ± 10.62	165.96 ± 29.50	174.21 ± 11.97	145 ± 53.52
**DYSPHNEA (+)**	0	30.1	81.2, *P*<0.001^§^	0
**PALPITATIONS (+)**	0	32.6 *P*<0.001^║^	68.8	28.6, *P*<0.001^║^
**HR (bpm)**	71.92 ± 9.50	87.04 ± 9.79	68.23 ± 11.00	71.33 ± 6.68
**SBP (mmHg)**	127.42± 17.02	128.63 ± 13.12	133.08 ± 11.41	121.33 ± 12.06
**DBP (mmHg)**	70.29 ± 12.41	77.04 ± 10.92	83.22 ± 7.39	76.00 ± 13.43
**LVEF (%)**	66.81 ± 7.17	45.20 ± 12.40*	47.21 ± 12.00†	57.71 ± 5.64
**TDLVD (mm)**	48.05 ± 4.68	55.94 ± 8.99	56.98 ± 8.65	47.98 ± 7.86
**TSLVD (mm)**	32.20 ± 6.17	1437.65 ± 10.26	42.96 ± 10.18	32.40 ± 5.97
**TAPSE RV (cm)**	21.58 ± 3.12	21.33 ± 3.23	21.35 ± 4.27	21.74 ± 1.22
**LA Area (cm2)**	17.26 ± 2.31	18.24 ± 4.32	19.80 ± 3.40	15.12 ± 4.50
**RA Area (cm2)**	13.67 ± 3.04	14.56 ± 3.97	16.11 ± 3.87	12.12 ± 2.91
**LA length (mm)**	48.02 ± 4.82	52 ± 9.07	60.59 ± 6.03	44.24 ± 4.55^‡^
**RA length (mm)**	45.54 ± 7.08	45.99 ± 7.06	52.70 ± 5.35	41.67 ± 5.15
**E wave (m/s)**	0.79 ± 0.14	0.79 ± 0.18	0.75 ± 0.23	0.86 ± 0.20
**A wave (m/s)**	0.55 ± 0.25	0.66 ± 0.22	0.70 ± 0.25	0.55 ± 0.14
**E/A**	1.34 ± 0.39	1.33 ± 0.45	1.14 ± 0.39	1.67 ± 0.60
**A septal**				
**Stdi (cm/s)**	7.87 ± 1.483	7.82±1.43	7.5 ± 01.50	8.45 ± 1.11
**Etdi**	8.72 ± 2.586	9.18±2.78	8.06 ± 1.64	11.40 ± 3.37
**Atdi**	7.68 ± 2.609	9.49±2.11	10.36 ± 1.85	7.72 ± 1.45
**A lateral**				
**Stdi**	10.40 ± 2.55	10.19 ± 2.46	9.81 ± 2.49	10.94 ± 2.38
**Etdi**	11.92 ± 4.48	12.90 ± 4.59	11.17 ± 3.23	16.35 ± 5.17
**Atdi**	9.14 ± 3.03	10.24 ± 2.34	10.18 ± 2.32	10.34 ± 2.58
**Fibrosis (+)**	0	26.5**^¶^**	62.5	28.6^£^
**Knock (+)**	0	30.5	43.8	42.9

BAG3 mutation carriers were divided into phenotypically negative (phenot -) or positive (phenot+) based on the presence of dysphnea and left ventricle disfunction.

Abbreviations: HR, heart rate; SBP, systolic blood pressure; DAP, dyastolic blood pressure; LVEF, left ventricle ejection fraction; TDLVD, telediastolic left ventricle diameter; TSLVD, telesistolic left ventricle diameter; TAPSE RV, tricuspid anular plane sistolic exceursion of the right ventricle; LA Area, left atrium area; RA area, right atrium area; Fibrosis +, presence of fibrosis; Knock +, presence of knock. * *P*<10^−4^ LVEF BAG3-/DCM- vs BAG3-/DCM+. **†** *P*<4x10^−3^ LVEF BAG3-/DCM+ vs BAG3+/DCM+. ‡ *P*<6x10^−3^ LA LENGHT BAG3-/DCM+ vs BAG3+/DCM+. **^§^** *P*<0.001 DYSPHNEA BAG3-/DCM+ vs BAG3+/DCM+. ║ *P*<0.001 PALPITATIONS BAG3-/DCM+ vs BAG3+/DCM+ AND BAG3+/DCM+ vs BAG3+/DCM-. **^¶^** *P*<0.001 PALPITATIONS BAG3-/DCM+ vs BAG3+/DCM+. **^£^** *P*<0.001 PALPITATIONS BAG3+/DCM+ vs BAG3+/DCM-.

### BAG3-related FDCM is associated with changes in the expression of circulating miRNAs

To first determine the miRNA profile associated to BAG3 mutation, the analysis of 1759 circulating miRNAs was performed in BAG3 mutant carriers (BAG3+/DCM+ and BAG3+/DCM-) and BAG3 wild-type individuals (BAG-/DCM+ and BAG3-/DCM-). By applying a criterion of 2-fold difference in the expression between groups, mir-3191-3p, -6769b-3p, -1249-ep, -154-5p, -6855-5p, and -182-5p were increased in BAG3+ mutant carriers (Figure 1C). A further analysis between BAG3-associated DCM (BAG3+/DCM+) versus BAG3 asymptomatic patients (BAG3+/DCM-) revealed no differences between miRNAs mir-3191-3p, 6769b-3p, and 1249-ep, while the levels of miRNAs mir-6855-5p, 182-5p, and 154-5p discriminated BAG3 symptomatic DCM versus BAG3 asymptomatic DCM patients (Figure 1B), as also shown when plotted the selected three miRNAs in a clustered heat map (Figure 1C).

A more detailed analysis did show a significant increase of main mir-154-5p and mir-182-5p levels (4.5 and 1.4 times, respectively) in BAG3+/DCM+ individuals (Figure 2A: BAG3+/DCM+ (DCM) vs BAG3+/DCM- (Control)), while mir-6855-5p was 2.3 times overexpressed in BAG3+/DCM- patients (Figure 2A). By contrast, no significant differences were found in the main expression of the same miRNAs in BAG3-/DCM+ versus BAG3-/DCM- individuals (mir-154-5p P: 0.9263; mir-182-5p P:0.403; mir-6855-5p P: 0.468). No gender differences were detected between DCM+ and DCM- patients, and the same applies when comparing clinical parameters, including LVEF (<50%: DCM+) (Figure 2B,C, respectively). Taken together, our data suggest that miRNAs mir-154-5p, -182-5p, and -6855-5p are specific of this type of FDCM.

**Figure 2:** Expression of selected miRNAs in the population study (**A**) Differential expression of mir-154-5p (left), mir-182-5p (middle), and mir-6855-5p (right) in BAG3+/DCM+ patients (DCM) compared with asymptomatic BAG3+/DCM- individuals (Control). (Mean ± SD, *P<0.05 mir-154-5p DCM vs Control. *P<0.01 mir-182-5p DCM versus Control. *P<0.01 mir-6855-5p DCM versus Control). (**B**) Differential expression of mir-154-5p, mir-182-5p, and mir-6855-5p in males (M) and females (F) BAG3+/DCM+ patients (DCM) compared with males (M) and females (F) BAG3+/DCM- individuals (C)). (*n*=21 Mean ± SD). (**C**) Differential expression of mir-154-5p, mir-182-5p, and mir-6855-5p between males and females with decreased LEVF (LVEF<50%).

### Association between BAG3-mediated DCM circulating miRNAs and severity of disease

We compared selected miRNA expression levels with the clinical parameters of the study (Table 1). When data were not stratified, negative correlations between systolic (*r* = −6059, *P*<0.006) and diastolic blood pressure (*r = −*4493, *P*<0.05), aortic diameter (*r* = −0.47179, *P*<0.003), left atrium length (*r* = −0.73897 *P*<0.0002), and left atrium area (*r* = 0.44648, *P*<0.05) with mir-6855-5p; and a positive correlation between A wave and mir-182-5p (*r* = 0.4908, *P*<0.002) were detected (Table 2). However, no statistical correlations were found between selected miRNAs and clinical prognostic parameters of disease, including LVEF or systolic and diastolic ventricular diameters (TDLVD, TSLVD).

**Table 2:** Pearson’s correlation coefficient between selected miRNAs and clinical parameters

	mir-6855-5p	mir-154-5p	mir-182-5p
**SBP**	*r* = −0.60592/*P*<0.006	*r* = −0.26238/*P*:0.291	*r* = −0.32274/*P*:0.1894
**DBP**	*r* = −0.44933/*P*<0.05	*r* = −0.23790/*P*:0.340	*r* = −0.17245/*P*:0.4926
**AOD**	*r* = −0.47179/*P*<0.05	*r* = −0.05152/*P*:0.8291	*r* = −0.24271/*P*:0.3017
**LAL**	*r* = −0.73897/*P*<0.0002	*r* = −0.10632/*P*:0.6552	*r* = −0.14169/*P*:0.5283
**LAA**	*r* = 0.44648/*P*<0.05	*r* = −0.4176/*P*:0.073	*r* = −0.31634/*P*:0.1811
**AW**	*r* = −0.40383/*P*:0.07	*r* = 0.11519/*P*<0.6283	*r* = 0.49081/*P*<0.05

The data shown above, lead us to investigate BAG3 associated DCM by gender and age stratification. Although the study did not show sex differences in the main levels of selected miRNAs (Figure 2B,C), when performing correlation analysis, positive statistical correlation in women BAG3+/DCM+ between LVEF, TDLVD, and TSLVD with selected miRNAs were detected (Table 3). By contrast, correlations were restricted to TDLVD with hsa-mir-6855-5p, and to LVEF with hsa-mir-182-5p in men younger than 40 years of age (Table 3). Besides, BAG3+/DCM- men or women did not show any statistical correlation between selected miRNAs and the clinical parameters of the study. Taken together these results suggest that selected miRNAs may forecast BAG3 associated FDCM between men and women.

**Table 3:** Pearson’s correlation coefficient between selected miRNAs and clinical parameters

	mir-6855-5p	mir-154-5p	mir-182-5p
**FEMALE**			
**LVEF**	*r* = 0.81513/ *P*<0.001	*r* = −0.21378/ *P*:0.1354	*r* = 0.8942/*P*<0.04
**TDLVD**	*r* = −0.9853/*P*<0.001	*r* = 0.18190/ *P*:0.08	*r* = −0.08267/*P*:0.364
**TSLVD**	*r* = −0.9859/*P*<0.02	*r* = 0.9952/*P*<0.001	*r* = −0.91862, *P*:0.06
**MALE**			
**LVEF**	*r* = −0.0470/*P*:0.08	*r* = 0.38182/*P*:0.08	*r* = 0.8710/*P*<0.04
**TDLVD**	*r* = −0.9970/*P*<0.04	*r* = −0.37954/*P*:0.11	*r* = −0.32413/*P*:0.163
**TSLVD**	*r* = 0.28112/*P*:0.06	*r* = −0.36242/ *P*:0.665	*r* = −0.359/*P*:

### The panel of mir-154-5p and mir-182-5p may forecast DCM in BAG3 mutant carriers

To further study the potential use of selected miRNAs as diagnostic tools, we compared the number of BAG3+/DCM+ patients, and healthy controls expressing a combination of two (double+) or three miRNAs. We found no differences between individuals co-expressing mir-154-5p and mir-6855-5p, neither subjects co-expressing mir-6855-5p and mir-182-5p (Figure 3A,B). By contrast, 56% of BAG3+/DCM+ individuals, significantly co-expressed both mir-154-5p and mir-182-5p, and a slight 4% did not, whereas on the opposite, no BAG3+/DCM- individuals co-expressed both miRNAs and 28% of them did not express any miRNA (double-) (Figure 3C), suggesting that the combination of mir-154-5p and mir-182-5p may potentially have diagnostic value.

**Figure 3:** Co-expression of selected miRNAs in the population study Percentage of BAG3+DCM-(Control) or BAG3+DCM+ (DCM) subjects, co-expressing two selected miRNAs (**A**) mir-154-5p/mir-6855-5p. (**B**) mir-6855-5p/mir-182-5p. (**C**) mir-154-5p/mir-182-5p. *n*=20, Mean ± SD. *P<0.01 Double + mir-154-5p/mir-182-5p DCM versus Control. ^$^*P*<0.01 Double - mir-154-5p/mir-182-5p DCM versus Control.

We used a ROC curve to test the accuracy of the results measured by the AUC to analyze co-expression of mir-6855-5p and mir-154-5p (Figure 4A), mir-6855-5p and mir-182-5p (Figure 4B), or mir-154-5p and mir-182-5p (Figure 4C), detecting a 74% accuracy (AUC), and a 84.6% sensitivity when using co-expression of mir-154-5p and mir-182-5p in BAG3/DCM patients (Figure 4C). Nevertheless, additional studies aimed to increase sample size should be performed for further validation.

**Figure 4:** Receiver operating characteristic (ROC) curves to test accuracy of selected miRNAs in the population study Diagnostic sensitivity and specificity of using the combination of mir-6855/mir-154 (**A**) mir-6855/mir-182 (**B**) and mir-154/mir-182 (**C**) delimited by ROC/AUC analysis.

## Discussion

In the present study, we currently report the differential expression of selected miRNAs in BAG3 deletion carriers from a small cohort of Spanish familial individuals with DCM. Among the 1759 miRNAs analyzed, significant differences between BAG3 mutants versus BAG3 wild-type individuals were found for mir-3191-3p, mir-6769b-3p, mir-1249-ep, mir-154-5p, mir-6855-5p, and mir-182-5p. Interestingly, DCM patients expressing BAG3 mutation differentially expressed mir-154-5p, mir-6855-5p, and mir-182-5p, when compared with asymptomatic BAG3 mutation carriers. The expression of selected miRNAs correlated with several parameters of disease, including blood pressure, left atrium area and length, while sex and age differences were found associated between selected miRNAs and diagnostic DCM parameters, including LVEF, TDLVD, and TSLVD. The combination of mir-154-5p and mir-182-5p, may have a predictive value of disease, since almost a 60% of BAG3+/DCM+ patients, co-expressed mir-154-5p and mir-182-5p, while a slight 4% did not expressed any miRNA.

Familial DCM counts for more that 50% of all cases reported of DCM, and most of them are associated with genetic variations of single genes including, ACTC1, RBM20, MYBPC3, MYH6, MYH7, TNNT2, TPM1, SCN5A, FHOD3, SLC39A8, MLIP, ALPK3, or BAG3 [2,22]. However, the transition between single point mutations and DCM still require further investigation. We and others have reported the relevance of BAG3 in the onset and progression of DCM [1,7,8,24,25,26]. BAG3 regulates myocyte contraction through interaction with L-type calcium channels [27], thus BAG3 mutations have been associated with different forms of familial cardiomyopathy, including DCM. Here, we provide new evidence which may help to explain the effect of BAG3 on DCM, by regulating the levels of selected miRNAs.

The implication of circulating miRNAs in the pathogenesis and progression of DCM in mice and in humans is well documented. Down-regulation of mir-1, mir-669a, mir-451a, and up-regulation of mir-3135b, mir-3908 and mir-5571-5p are related with DCM progression [20,28]. Recently it was found a correlation between the time by which selected miRNAs are expressed and beta-blocker administration induces reverse remodeling in DCM patients [29], but the relationship between BAG3-mutation carriers with DCM and the expression profile of miRNAs remains unknown. Here, we show that DCM patients carrying a BAG3-mutation show differential expression of mir-6855-5p, mir-182-5p, and mir-154-5p.

miRNA mir-182 family members play a role in cardiovascular disease, including myocyte hypertrophy [30], heart failure [31], and cardiac allograft rejection [32,33]. On the other hand, mir-154 inhibition reduces cardiac fibrosis, cardiac myocyte size, and cardiac dysfunction [34]. With regard to the expression of mir-6855-5p, we describe here for the first time the relationship between BAG3-mutation carriers with DCM and systolic (*r* = −6059, *P*<0.006), diastolic blood pressure (*r* = −4493, *P*<0.05), aortic diameter (*r* = −0.47179, *P*<0.003), left atrium length (*r* = −0.73897, *P*<0.0002), and left atrium area (*r* = 0.44648, *P*<0.05). Interestingly, we found sex differences in the relationship between mir-6855-5p with LVEF (*r* = 0.81513, *P*<0.001), TELVD (*r* = −0.9853, *P*<0.001), and TSLVD (*r* = −0.9859, *P*<0.02) in women, while in men mir-6855-5p statistical correlation was restricted to TDLVD (*r* = −0.9970, *P*<0.04).

Targets of mir-182-5p may include genes encoding for several transcription factors, cell cycle regulators and apoptosis related proteins, including Bcl2 [35]. As part of the mechanism induced to prevent heart failure and ischemia/reperfusion damage, BAG3 promotes cell survival through binding to several proteins including hsp70 and Bcl2 [36]. In DCM BAG3-mutation carriers, the levels of mir-182-5p resulted significantly elevated respect to asymptomatic patients, and correlated with LVEF both in men and women, suggesting that lack of mir-182-5p expression may be related with the antiapoptotic effect of BAG3 in the heart, as others reported in mice overexpressing BAG3, and subjected to myocardial infarction, showing improved left ventricular function, and reduced hypoxia-induced cardiomyocyte apoptosis [37].

Statistical correlation was found between mir-154-5p and TSLVD in DCM female BAG3+ patients. Important targets of mir-154-5p may include Dicer, which on its absence induces significant DCM in mice, and is considerably abundant in patients with LV assistant devices to improve cardiac function [25]. Other targets may also include Wnt11, in which mir-154-5p targets Wnt11 during osteogenic differentiation [32] and improves cardiac function in Coxsackievirus induced myocarditis [38], and DiGeorge syndrome [33], but the specific role of mir-154-5p on Wnt11 in DCM is still unknown.

Almost 60% of BAG3+/DCM+ patients co-expressed a combination of mir-182-5p, and mir-154-5p, and ROC/AUC analysis evidenced a significant level of confidence and accuracy. Considering the significant limitations of the study (reduced sample size, lack of follow-up analysis of patients and lack of miRNA derived target genes), our data suggest that the combination of mir-154-5p and mir-182-5p may potentially have diagnostic value of FDCM.

Average age of BAG3+/DCM- group patients was 26 years old, another significant limitation of the study. Therefore, further analyses focused to reduce the above limitations, will shed light about future diagnostic value of selected miRNAs found in the present study.

## Summary

- The culprit genes underlying the pathogenesis of more than 50% of familial DCM are still unknown.
- A new FDCM associated to mutation in the BAG3 gene was detected. DCM positive family members differentially express selected miRNAs depending on BAG3 expression. Statistical correlations between selected miRNAs and DCM critical parameters were found.
- Our data suggest that the combination of selected miRNAs may potentially have a diagnostic value of FDCM. Considering the significant limitations of the study (reduced sample size, lack of follow-up analysis of patients and lack of miRNA derived target genes), further investigations focused to reduce the above limitations will shed light about implementation in the population.

## Abbreviations

AUC: area under the ROC curve
BAG3: Bcl2-associated athanogene 3
DBP: dyastolic blood pressure
ECG: electrocardiogram
FDCM: familial dilated cardiomyopathy
Fibrosis +: presence of fibrosis
HR: heart rate
Knock +: presence of knock
LA area: left atrium area
LEVF: left ventricle ejection fraction
miRNA: microRNA
RA area: right atrium area
ROC: receiver operating characteristic
SBP: systolic blood pressure
TAPSE RV: tricuspid anular plane sistolic exceursion of the right ventricle
TDLVD: telediastolic left ventricle diameter
TSLVD: telesistolic left ventricle diameter
